The article "Brain-derived exosomes from dementia with Lewy bodies propagate α-synuclein pathology" was retracted in 2026. Reasons: duplicated images; duplicated data; overlap with earlier publications; unreliable data.

# Brain-derived exosomes from dementia with Lewy bodies propagate α-synuclein pathology

**DOI:** 10.1186/s40478-017-0445-5

**Published:** 2017-06-09

**Authors:** Jennifer Ngolab, Ivy Trinh, Edward Rockenstein, Michael Mante, Jazmin Florio, Margarita Trejo, Deborah Masliah, Anthony Adame, Eliezer Masliah, Robert A. Rissman

**Affiliations:** 1 Department of Neurosciences, UCSD School of Medicine, La Jolla, CA 92093 USA; 2 Department of Pathology, UCSD School of Medicine, La Jolla, CA 92093 USA; 3 Veterans Affairs San Diego Healthcare System, San Diego, CA 92161 USA

**Keywords:** Alzheimer’s disease, Exosomes, Alpha synuclein, Lewy body, Tau, Amyloid beta, Dementia

## Abstract

Proteins implicated in neurodegenerative conditions such as Alzheimer’s disease (AD) and Dementia with Lewy Bodies (DLB) have been identified in bodily fluids encased in extracellular vesicles called exosomes. Whether exosomes found in DLB patients can transmit pathology is not clear. In this study, exosomes were successfully harvested through ultracentrifugation from brain tissue from DLB and AD patients as well as non-diseased brain tissue. Exosomes extracted from brains diagnosed with either AD or DLB contained aggregate-prone proteins. Furthermore, injection of brain-derived exosomes from DLB patients into the brains of wild type mice induced α-synuclein (α-syn) aggregation. As assessed through immunofluorescent double labeling, α-syn aggregation was observed in MAP2^+^, Rab5^+^ neurons. Using a neuronal cell line, we also identified intracellular α-syn aggregation mediated by exosomes is dependent on recipient cell endocytosis. Together, these data suggest that exosomes from DLB patients are sufficient for seeding and propagating α-syn aggregation in vivo.

## Introduction

Misfolded protein aggregates are a pathological hallmark of age-related neurodegenerative disorders such as Alzheimer’s disease (AD) and Dementia with Lewy Bodies (DLB) [7, 26]. Termed proteinopathies, both disorders result in synaptic dysfunction, neuron loss and cognitive decline [2, 26]. AD pathology is classically defined as plaques composed of amyloid beta (Aβ) and neurofibrillary tangles containing tau [13]. Likewise, Lewy Body disorders such as DLB are characterized by clusters of α-synuclein (α-syn) within the neuron cell body (called “Lewy Bodies”) and terminals [36]. Yet the brains of patients clinically diagnosed with either disorder also contain other aggregate formations. For example, Aβ plaques are present in patients diagnosed with Lewy Body disorders, with DLB plaque loads comparable to AD [14, 20, 22, 44]. Conversely, patients with the “plaque-only” variant of AD contain Lewy Bodies within the neocortex and brainstem [13, 21]. Such heterogeneity between AD and DLB obfuscates proper treatment and diagnosis*.*

The article "Brain-derived exosomes from dementia with Lewy bodies propagate α-synuclein pathology" was retracted in 2026. Reasons: duplicated images; duplicated data; overlap with earlier publications; unreliable data.

Aβ, Tau and α-syn are thought to reconfigure into a neurotoxic species that migrates into neighboring cells and triggers protein aggregation [4]. Studies investigating plaque initiation found Aβ plaques in animal brains intracranially injected with AD patient brain homogenates [1, 37]. Neurofibrillary tangles and Lewy Bodies were also seen in rodent brains injected with brains homogenates of tauopathy and synucleinopathy patients, respectively [10, 24]. The seeding of exogenous misfolded proteins initiated the aggregation of endogenous non-diseased protein, a characteristic similar to prion proteins involved in spongiform encephalopathy. In 2008, two separate studies reported α-syn-positive deposits in human fetal dopaminergic neurons grafted into Parkinson’s disease patients [25, 31]. Because α-syn aggregation is not observed in midbrain neurons until middle age [9], it was concluded that the implanted neurons acquired α-syn pathology through host-to-graft transmission. Subsequent studies in rodents and cell culture demonstrated neuron-to-neuron transfer of α-syn, another characteristic thought to be exclusive to prion proteins [12]. It is now accepted that Aβ, tau and α-syn possess the ability to self-propagate and utilize cellular connections to spread throughout the brain in a network-specific manner as observed in human patients and rodent models [4].

Although multiple methods of aggregate-prone protein transmission have been proposed, such as the formation of microtubes and membrane shedding, one attractive mechanism of protein aggregate spread is through exosomes [3, 30, 42, 45]. Originating inside multivesicular bodies (MVB) of the endocytic pathway, exosomes are 40–100 nm vesicles that are released into the extracellular space through the fusion of a MVB to the plasma membrane [27]. Originally thought to serve as an alternative method of waste elimination, exosomes participate in the transmission of various proteins and RNA between cells [17]. Interestingly, α-syn, tau and amyloid precursor protein (APP) are present within exosomes in vitro [11, 15, 41, 43, 53]. Exosomes harboring neurodegenerative-associated proteins have been detected in blood, CSF and urine of patients with neurodegenerative diseases [51]. Importantly, exosomes extracted from the plasma of MCI and AD patients induced the formation of tau pathology in non-diseased mice [53]. While CSF derived exosomes from DLB patients have initiated α-syn aggregation in vitro [47], it is unknown whether exosomes derived from DLB patients exhibit similar pathogenicity in vivo.

The article "Brain-derived exosomes from dementia with Lewy bodies propagate α-synuclein pathology" was retracted in 2026. Reasons: duplicated images; duplicated data; overlap with earlier publications; unreliable data.

The aims of this study were to 1) determine if the protein content of brain-derived exosomes from patients diagnosed with AD or DLB contain Aβ, tau and/or α-syn over non-diseased individuals and 2) test the hypothesis that brain derived exosomes from DLB patients can seed and propagate α-syn pathology. Utilizing biochemical techniques and animal models, we show that brain exosome cargo isolated from AD and DLB brain tissue contain Aβ and tau, with exosomes derived from DLB brain tissue specifically containing α-syn. Furthermore, administering brain-derived exosomes into the brains of non-diseased mice induced α-syn aggregates in neurons, further bolstering the hypothesis that neurotoxic proteins such as α-syn can be packaged into exosomes to exacerbate synucleinopathy. Lastly, we demonstrate that α-syn aggregation triggered by DLB exosomes is dependent on endocytosis. These data further emphasize the role of exosomes in propogating DLB pathology.

## Materials and methods

### Human samples

The demographics and diagnoses presented in Table 1 were obtained from patients neurologically and psychometrically studied at the Alzheimer Disease Research Center (ADRC) University of California, San Diego (UCSD). All procedures were reviewed and approved by the UCSD Institutional Review Board. Upon autopsy, patient brains were collected by the UCSD ADRC Neuropathology Core and sagittally divided at autopsy; the left hemibrain was fixed in 10% buffered formalin for neuropathological analysis and the right frozen at −70 °C for subsequent exosome isolation.

**Table 1:** Summary of clinical and pathological characteristics of all donors

Diagnosis	Age (years)	Brain weight (g)	Education (years)	DRS	Braak stage	Plaques (counts/0.1 mm^2^)	Tangles (counts/0.01 mm^2^)	Amyloid angiopathy (score)	Lewy bodies (score)
Ctl (*N* = 3)	82.33 ± 5	1142 ± 111	14 ± 3.4	140 ± 1	0	4.67 ± 0.67	0	0	0
AD (*N* = 3)	81.3 ± 4.7	1100 ± 156	12 ± 0	72.7 ± 8.3	6.2 ± 0	47.3 ± 4.6	6.7 ± 4.2	3	0
DLB (*N* = 3)	77 ± 13.9	1237 ± 9.7	14.7 ± 3.1	104 ± 11	4.2 ± 2.8	33 ± 1	2 ± 1	0.7 ± 0.2	3

Values reported in table are expressed as arithmetic mean ± standard mean of error (SEM)

*Abbreviations*: *AD* Alzheimer’s Disease, *Ctl* Control, *DBL* Dementia with Lewy Bodies, *DRS* Mattis Dementia Rating Scale

### Ultracentrifugation

Exosomes were isolated from frozen brain tissue (Fig. 1a) as previously described [40]. Briefly, 0.5 g of frozen frontal cortex was dissected and immersed in a solution of 20 units/ml of papain in Hibernate E (Life Technologies) (10:1 ratio) for 15 min at 37 °C. About 20 ml of cold Hibernate E was added before homogenization. The brain homogenate was passed through a 40 μl mesh filter then fractionated though differential centrifugation: 300 *g* for 10 min, 2000 *g* for 10 min, 10,000 *g* for 30 min. The resulting supernatant was further clarified using a 0.2 μm mesh filter and then centrifuged at 100,000 *g* for 70 min at 4 °C. The pellet was washed twice in 5 ml PBS prior to centrifugation at 100,000 *g* for 80 min. Both the supernatant (“control fraction”) and pellet (“exosome fraction”) were collected for further analysis. Antibodies towards CD63 (Systems Bioscience, Cat. No: EXOAB-CD63A-1), CD81 (Systems Bioscience, Cat. No: EXOAB-CD81A-1) and Alix (3A9, BioLegend, Cat. No:634,501) were used to characterize each fraction.

The article "Brain-derived exosomes from dementia with Lewy bodies propagate α-synuclein pathology" was retracted in 2026. Reasons: duplicated images; duplicated data; overlap with earlier publications; unreliable data.

**Fig. 1:** Isolation of exosomes from patient brain tissue. **a** Schematic of ultracentrifugation protocol used to isolate exosomes from tissue. Note that the pellet is the “exosome fraction”, and the supernatant is the “control fraction”. **b** Exosome identification markers present in the exosome fraction of Ctl, AD and DLB brain tissue. **c** *Top Row:* Representative EM micrographs from control fraction as well as Ctl, AD and DLB exosome fractions. *Bottom Row:* EM micrographs from control fraction and Ctl, AD and DLB exosome fractions stained with immunogold labeled anti-CD 63. Scale bar = 50 nm

### Mice

Rodent experiments abided with NIH recommendations for good animal practice and all animal use procedures were reviewed and approved by the UCSD Institutional Animal Care and Use Committee. Male C57BL/6 N × DBA/2 F1 mice, ~4 months old, were intracranially injected with exosomes derived from a DLB patient (*N* = 6) or a non-diseased patient (*N* = 5). 4.4 μg (~2 μl in volume) of the exosome fraction was sterotaxically injected into hippocampus (−2.0 AP, +1.5 ML, −1.3 DV) [39]. Four weeks post injection, mice were anesthetized with chloral hydrate (Sigma, C8383) and transcardially perfused with 0.9% saline. Brains were removed and drop-fixed in phosphate-buffered 4% paraformaldehyde, pH 7.4, at 4 °C for 48 h for further analysis.

### Immunohistochemistical analysis

Paraffin sections from 10% buffered formalin-fixed human neocortical, limbic system and subcortical material were stained with hematoxylin and eosin, thioflavin S, ubiquitin (Dako, Z0458) and α-syn (Millipore, AB5038P) were used for routine neuropathological analysis that included assessment of plaques, tangles, Lewy bodies and Braak stage. Additional staining for Syn1 (BD Biosciences, Cat. No: 620,787), phosphorylated α-syn at serine 129 (pSer129 α-syn, Abcam, Cat.No: ab51253), Aβ (4G8, Covance, Cat. No: SIG-39200; 6E10, Covance, Cat.No: SIG-39320) and pTau^396^ (antibody PHF1, generous gift from Dr. P. Davies) were performed to further characterize Aβ and tangle protein composition. Mouse brains injected with human brain-derived exosomes were serially sectioned at 40 μm (Vibratome 2000, Leica, Wetzlar, Germany). Free-floating sections relevant to the injection site were incubated overnight at 4 °C with Syn1 antibody, followed by biotinylated horse anti-mouse IgG (1:100; Vector Laboratories, BA-1000), Avidin D-horseradish peroxidase (1:200; Vector Laboratories, A-2004), and subsequent detection with diaminobenzidine (DAB, Vector Laboratories, SK-4100). Sections were imaged with a bright-field digital microscope (Olympus, Shinjuku, Japan). Counts of Syn1, pSer129 α-syn, Aβ and PHF1 immunoreactivity were performed using Image J and expressed as optical density. A total of four images per group were captured, converted to gray scale, processed for proper threshold and dynamic scale set to determine optical density.

The article "Brain-derived exosomes from dementia with Lewy bodies propagate α-synuclein pathology" was retracted in 2026. Reasons: duplicated images; duplicated data; overlap with earlier publications; unreliable data.

### Immunofluorescent colocalization analysis

For the double labeling studies, 40 μm sections were immunolabeled with the Syn1 antibody and either MAP2 (Clone 2B, Millipore, Cat. No: MAB378), Rab5 (15/Rab5, BD Biosciences, Cat. No: 610,281), GFAP (Millipore, Cat. No: MAB3402) or a mouse specific α-syn antibody (a generous gift from V.M-Y. Lee). Human α-syn immunoreactivity was detected with a FITC-tagged secondary antibody (Vector), while the other antibodies were visualized with the Tyramide Signal Amplification™-Direct (Red) system (Perkin Elmer). All sections were processed simultaneously under the same conditions, and experiments were performed in duplicate in order to assess the reproducibility of results. All fluorescent imaging studies were done on a DMI 4000B inverted fluorescent microscope (Leica, Germany) with an attached TCS SPE confocal system (Leica), using a Leica 63X (N.A. 1.3) objective. A total of four optically paired micrographs were analyzed with ImageJ colocalization color map plugin to determine the percent of human α-syn positive clusters within Rab5, MAP2, and GFAP expressing cells. Efficacy of of α-syn cross-seeding was reported as percent mouse α-syn clusters detected within human α-syn positive cells.

### Western blot

Protein content from exosome and control fractions was separated on 4–12% Bis-Tris gels (Life Technologies, NP0322BOX) then transferred to a polyvinylidene fluoride (PVDF) membrane (Immobilon-P, Millipore, IPFL00010). The membrane was blocked in 1% *w*/*v* BSA in PBS with 0.1% Tween 20 (PBS-T) for 1 h at room temperature, followed by overnight incubation in primary antibody at 4 °C. Primary antibodies listed in the immunohistochemistry section above to were used to characterize exosome protein cargo. After washing with PBS-T, the membrane was incubated in the dark with HRP-conjugated secondary antibodies specific to the primary antibody host for 1 h at room temperature. Protein bands were detected using Pierce ECL Plus Western Blotting substrate (Thermo Scientific, 32,134) through a BioRad Molecular Imager ChemiDoc (BioRad, Hercules, CA).

The article "Brain-derived exosomes from dementia with Lewy bodies propagate α-synuclein pathology" was retracted in 2026. Reasons: duplicated images; duplicated data; overlap with earlier publications; unreliable data.

### Transmission electron microscopy

To characterize exosomes, pellets fraction were fixed in the ultracentrifugation tube with 4% PFA for 30–60 min at room temperature. Pellet post-fixation was performed with 1% OsO_4_ for 30 min and then rinsed with distilled water. Following graded ethanol dehydration, the pellet was block-stained with 1% uranyl acetate in 50% ethanol for 30 min. The pellet was embedded in Taab 812 (Taab; Aldermaston, UK) and polymerized for 12 h at 60 °C. 50–60 nm ultrathin sections were cut using a Leica UCT ultramicrotome (Leica Microsystems, UK) and examined using a Hitachi 7100 transmission electron microscope (Hitachi Ltd., Japan). Electron micrographs were taken by a Veleta 2 k × 2 k MegaPixel side-mounted TEM CCD camera (Leica Microsystems). Contrast/brightness of electron micrographs was edited using Adobe Photoshop CS3.

To visualize the presence of α-syn within intact exosomes, fixed exosome pellets were blocked with exosome FSGB buffer (5% FSGB, 5% BSA in 50 mM Tris/HCl pH 7.4) and incubated with Syn1 or CD63 (1:100 diluted in 1% FSGB and 1% BSA in PBS) overnight at 4 °C. After washing, pellets were incubated with secondary antibody (goat anti mouse IgG 6 nm gold particles 1:80, AURION 806.022 diluted in 0.2% BSA in PBS) for 2 h. Exosome pellets were washed with 0.2% BSA in PBS and then with PBS alone. After post-fixation in 1% glutaraldehyde for 10 min, the pellets were washed 2 times with distilled water and processed for visualization as described above.

### Cell culture

The B103 rat neuroblastoma cell line was used to visualize exosome-mediated α-syn uptake due to previous observations of α-syn overexpression triggering excessive intracellular oligomeric α-syn accumulation and neurite growth reduction [50]. Cells were seeded at 5 × 10^4^ cells per well on poly-L-lysine coated glass coverslips contained in a 12-well plate 24 h prior to exosome incubation. Endosomal inhibition was performed either by incubating cells in 4 °C for 30 min or treating with 80 μm Dynasore, a dynamin GTPase inhibitor, dissolved in DMSO for 30 min at 37 °C.

### Statistical analysis

All microscopic quantifications were performed blind-coded with four fields per slide evaluated per group. All values in the figures are expressed as arithmetic mean ± standard mean of error (SEM). Differences in optical density and percent colocalization between Ctl and DLB groups were analyzed using the two-tailed unpaired Student’s *t*-test. Statistical analyses were calculated using Prism (GraphPad Software).

The article "Brain-derived exosomes from dementia with Lewy bodies propagate α-synuclein pathology" was retracted in 2026. Reasons: duplicated images; duplicated data; overlap with earlier publications; unreliable data.

## Results

### Cohort clinicopathological data

Table 1 summarizes the clinical and pathological data of each cohort. Tissue samples were from age-matched non-diagnosed (Ctl) as well as AD or DLB individuals (*N* = 3/cohort). There were no significant differences in age or brain weight between groups. Patients diagnosed with either AD or DLB scored below Ctl individuals in the Mattis Dementia Rating Scale (DRS) (Ctl: 140 ± 1, AD: 72.7 ± 8.3, DLB: 104 ± 11), a test used to determine cognitive decline [35]. Each cohort received at least 12 years of education, as number of years of education has shown to impact DRS performance (Ctl: 14 years ±3.4, AD: 12 years ±0, DLB: 14.7 years ±3.1) [8]. The AD and DLB brain tissues were scored in the later Braak stages (AD: 6.2 ± 0, DLB: 4.2 ± 2.8), while Ctl tissue did not exhibit any prominent Braak stage characteristics (Ctl:0). Plaque density was greater in AD and DLB patient tissue compared to Ctl tissue (Ctl: 4.67 ± 0.67, AD: 47.3 ± 4.6, DLB: 33 ± 10). Similarly, neurofibrillary tangle density was higher in AD and DLB patient tissue relative to Ctl tissue (Ctl: 0, AD: 6.7 ± 4.2, DLB: 2 ± 1). Aβ angiopathology was prevalent in patient brains from AD patients (Ctl: 0, AD: 3 ± 0, DLB: 0.7 ± 0.2) while Lewy Bodies were found exclusively in DLB brain tissue (Ctl: 0, AD:0, DLB: 3 ± 0).

### Exosomes isolated from brain tissue

Brain tissue from each cohort detailed in Table 1 was processed via ultracentrifugation to isolate brain-derived exosomes (Fig. 1a). The resulting pellets (“Exosome fraction”) and supernatant (“Control fraction”) from each cohort were analyzed by Western blot for tetraspanins CD63 and CD81 as well as the cytosolic protein Alix. These proteins are enriched in exosomal populations and are used to identify exosomes [32]. Exosome fractions of all cohorts expressed abundant amount of CD63, CD81 and Alix compared to Control fractions (Fig. 1b). TEM identified the presence of small vesicles in the exosome but not control fraction of all cohorts (Fig. 1c). Furthermore, immunogold staining for CD63 was present within the small vesicles in every exosomal fraction (Fig. 1c). These data verify that exosomes were successfully extracted from frozen brain tissue of healthy individuals as well as AD and DLB patients.

### Exosome cargo reflects brain pathology

We then assessed the cargo of brain-derived exosomes for aggregation-prone proteins. To further characterize the protein aggregates identified in Table 1, brain tissue from each cohort was analyzed for Aβ, tau and α-syn through immunohistochemical staining (Fig. 2a). Ctl tissue was negative for Aβ, tau and α-syn staining. AD tissue exhibited strong α-syn-positive clusters, Aβ plaques and dense p-Tau positive cell bodies. Brain tissue from DLB patients contained large α-syn positive intracellular deposits, indicative of LB formation, as well as positive Aβ staining. Western blot analysis revealed prominent signal for α-syn specifically in the DLB exosome fraction (Fig. 2b), while Aβ and p-Tau was present in both the AD and DLB exosome fraction (Fig. 2c-d). In summary, disease-associated proteins present in AD and DLB brain tissue were identified in their respective exosome fraction, consistent with previous studies assessing exosome content isolated from transgenic rodent brain tissue [40, 41].

The article "Brain-derived exosomes from dementia with Lewy bodies propagate α-synuclein pathology" was retracted in 2026. Reasons: duplicated images; duplicated data; overlap with earlier publications; unreliable data.

**Fig. 2:** Aggregate prone proteins associated with disease are present in exosome cargo. **a** Representative micrographs of Ctl, AD and DLB brain tissue, immunohistochemically stained for α-synuclein (α-syn), Amyloid Beta (Aβ) and phosphorylated tau (p-Tau). Scale bar for: α-syn = 5 μm, Aβ = 10 μm and p-Tau = 5 μm. **b**-**d** Western blots detecting the presence of α-syn (**b**), Aβ-protein (**c**) and p-Tau (**d**) contained within each fraction

### Brain derived exosomes from DLB patient facilitates α-syn accumulation

Previous studies have detected tau accumulation in mouse brain tissue upon intracranial injection of cerebral spinal fluid (CSF) exosomes derived from AD patients [53]. Could exosomes derived from DLB brain tissue exhibit similar properties and transmit DLB pathology to non-diseased tissue? To address this question, we injected exosome fractions extracted from Ctl and DLB human brain tissue into the cerebrum of non-diseased mice (Fig. 3b). TEM immunogold labeling detected visible α-syn clusters within exosomes from the DLB exosomal fraction (Fig. 3a). DLB-injected mouse brains exhibited significant intracellular and dendritic α-syn immunostaining around the injection site compared to Ctl-injected mouse brains (Fig. 3c, arrowheads, Fig. 3e). Higher levels of phosphorylated α-syn (pSer129 α-syn) staining were observed in DLB-injected brain tissue compared to Ctl-injected tissue (Fig. 3d, e). A significant amount of phosphorylated tau staining around the cell membrane was detected in DLB-injected tissue compared to Ctl-injected tissue; however, Aβ expression was low in both DLB and Ctl-injected groups (Fig. 3d, e).

**Fig. 3:** Administration of DLB exosomes into mouse brains initiates intracellular accumulation of phosphorylated proteins. **a** Representative EM micrographs of exosomes from Ctl and DLB brain samples immunolabeled for α-syn. **b** Schematic of stereotaxic injection into the hippocampus of C57BL/6 N × DBA/2 F1 mice. **c** Representative brightfield micrographs from mouse brains injected with control or DLB exosomes. *Row 1*: Sagittal view of the hippocampal area. Needle entry site is highlighted by arrowhead. Boxes highlight region of interest depicted in micrographs below. Scale bar = 150 μm. *Rows 2–3*: High magnification view of highlighted areas. Arrowheads highlight immunolabeled cell bodies. Scale bar = 25 μm. **d** Micrographs of brain tissue stained with phosphorylated α-syn (pSer129), PHF1 and Aβ (6E10). Scale bar = 25 μm. **e** Quantification of immunohistochemical stains from (**c**) and (**d**) through optical density. * = *P* < 0.05. Error bars indicate SEM

The article "Brain-derived exosomes from dementia with Lewy bodies propagate α-synuclein pathology" was retracted in 2026. Reasons: duplicated images; duplicated data; overlap with earlier publications; unreliable data.

### Accumulation of α-syn occurs in neurons and astrocytes

Next, we sought to further characterize the mechanisms DLB-derived exosomes utilize to potentially trigger α-syn pathology using immunofluorescent colabeling techniques. Significant amounts of colocalization of α-syn with Ras-related in brain 5 (Rab5), a small GTPase associated with the biogenesis of multivesicular bodies [5], occurred in DLB but not Ctl-injected brain slices (Fig. 4a, b). Additionally, brains administered with DLB derived exosomes expressed significantly higher levels of α-syn accumulation in MAP5^+^ cells in than Ctl, implicating DLB exosomes were internalized in neurons (Fig. 4c, d). Interestingly, α-syn clusters were present in GFAP^+^ cells of DLB-injected brain tissue when compared to Ctl (Fig. 4e, f). Finally, colocalization of human and mouse α-syn was exclusively detected in DLB injected brain slices (Fig. 4g, h). Taken together, these data suggest that exosomes harboring potentially pathogenic forms of α-syn can be taken up by non-diseased neurons and possibly astrocytes to induce α-syn accumulation.

**Fig. 4:** Human α-syn internalization occurs in neurons and astrocytes. Representative immunofluoresent micrographs of mouse hippocampal brain slices injected with either Ctl or DLB exosomes, depicting human α-syn (*Green*), DAPI (*Blue*) and **a** Rab5, **c** MAP2, **e** GFAP or **g** mouse α-syn (*Red*). Scale bar = 25 μm. Percent colocalization of α-syn and **b** Rab5, **d** MAP2, **f** GFAP and **h** mouse α-syn. * = *P* < 0.05. Error bars indicate SEM

### Exosome-mediated α-syn accumulation is mediated by endocytosis

Rab5 plays a broad role in the early endocytic pathway; one major process regulated by the small GTPase is endocytosis [5]. Previous studies suggest exogenous α-syn is endocytosed via Rab5, leading to the formation of LB and neuronal cell death [48]. To determine if DLB derived exosomes utilize endocytotic mechanisms, we implemented a cell-based assay to assess α-syn aggregation. First, to verify exosome content, exosome fractions from Ctl and DLB patients were characterized through Western Blot. Exosome markers CD63 and 81 were detected in both fractions and α-syn exclusively in the DLB fraction (Fig. 4a). In addition, EM analysis detected α-syn within DLB exosomes (Fig. 4b). A significant amount of α-syn particles were identified in B103 neuroblastomas incubated with DLB-derived but not Ctl exosomes (Fig. 4c, d). To determine if endocytosis regulated exosome internalization of α-syn, B103 neuroblastomas were incubated with either Ctl or DLB exosomes prior to endosomal inhibition either through 4 °C incubation or application of Dynasore. Dissociation of the microtubule complex involved in endocytosis by 4 °C incubation reduced the number of α-syn-positive particles (Fig. 4c, d). Similarly, inhibition of clathrin-mediated endocytosis through Dynasore diminished detection of α-syn-positive clusters (Fig. 4c, d). Together, these data further suggest that the internalization of exosomes originating from DLB patients via endocytosis promotes the intracellular aggregation of α-syn.

The article "Brain-derived exosomes from dementia with Lewy bodies propagate α-synuclein pathology" was retracted in 2026. Reasons: duplicated images; duplicated data; overlap with earlier publications; unreliable data.

## Discussion

Aggregate prone proteins are present in the biofluids of patients with synucleinopathies diseases [18, 19, 23, 28, 46]. However, it is unclear how exosomes are involved in transmitting synuclein pathology. Previously, CSF exosomes isolated from patients diagnosed with various synucleinopathies induced oligomerization of soluble α-syn in cell culture [47]. In this exploratory study, we demonstrate that viable exosomes containing Aβ, tau and α-syn isolated from patients clinically and pathologically diagnosed for DLB (Table 1, Figs. 1 and 2) can initiate α-syn and tau accumulation in non-diseased rodent brains (Fig. 3). In addition, human α-syn accumulation mediated by DLB exosomes was internalized in both mature neurons and astroglia (Fig. 4c-f). Finally, delivery of α-syn via exosomes was mediated by endocytosis (Fig. 5). These data provide additional insight to how exosomes can serve a vector for α-syn internalization and possibly take part in α-syn pathogenesis.

**Fig. 5:** Inhibition of endocytosis inhibits exosomes-mediated α-syn accumulation. **a** Immunoblot and **b** electron microscopy confirm the presence of α-syn containing exosomes from DLB patient. Scale bar = 50 nm. **c** B103 neuronal cell lines incubated with either Ctl or DLB exosomes and were left alone (*first row, Baseline*), incubated in 4 °C (second row) or incubated with Dynasore (*third row*). Accumulation of α-syn was visualized using the Syn1 antibody. Detail column indicates the region of interest magnified. **d** Quantification of α-syn positive particles in 37 °C (*baseline*), incubation at 4 °C and at 37 °C with Dynasore. * = *P* < 0.05 (DLB compared to Ctl). Error bars indicate SEM

Exosomal α-syn is detected in various bodily fluids of patients with Lewy Body disorders, yet the pathological potential is poorly understood [51]. Interestingly, individuals with Parkinson’s Disorder (PD) exhibited a significant decrease of total CSF α-syn and exosomes compared to controls [46, 47]. Even lower levels of CSF exosomes were detected in DLB patients compared to other synucleinopathy patients [47]. In this study, we further characterize the content of DLB derived exosomes and detect Aβ and tau within the cargo (Fig. 2c, d). Previous studies have shown Aβ interacts with α-syn to induce toxicity [34]. Although Aβ accumulation is not present in DLB-injected brain tissue, Aβ could interfere with the components involved in exosome biogenesis leading to overall exosome reduction. Despite the overall decrease in total exosomes, DLB CSF exosomes contained a greater amount of α-syn per exosome compared to PD CSF exosomes and incited α-syn aggregation [47]. We observed intracellular accumulation of phosphorylated α-syn and tau upon administration of DLB brain derived exosomes to healthy rodent brain tissue (Fig. 3d, e), providing additional evidence that DLB-derived exosomes have pathogenic potential. In addition, α-syn accumulation observed around the soma was of human origin (Fig. 4g), further suggesting DLB exosomes contained high levels of α-syn. It is important to note that we extract exosomes from frozen brain tissue via ultracentrifugation to enrich for brain-derived exosomes (Fig. 1a, [40]). It is possible that the exosome population assessed in our study may not reflect the exosomal population in the CSF. Nevertheless, understanding the properties of DLB exosomes could shed light into α-syn pathology. Furthermore, characterizing brain-derived exosomes may provide further information to distinguish central nervous system-derived exosomal populations in bodily fluids.

The article "Brain-derived exosomes from dementia with Lewy bodies propagate α-synuclein pathology" was retracted in 2026. Reasons: duplicated images; duplicated data; overlap with earlier publications; unreliable data.

Greater than 90% of LBs in patients with synucleinopathies contain α-syn phosphorylated at serine residue 129 (pSer129 α-syn) [38]. Furthermore, pSer129 α-syn is associated with dementia as higher levels are present in DLB than in PD [49]. Therefore, detecting pSer129 α-syn would provide insight into the pathogenicity of α-syn harbored in DLB exosomes. Indeed, prominent LBs were present in DLB patient tissues (Table 1, Fig. 2a). Importantly, a significant amount of pSer129 α-syn staining was quantified in DLB-injected brain tissue (Fig. 3d-e), implying that exosomes extracted from DLB brain tissue contained pSer129 α-syn. However, phosphorylation of human α-syn is thought to occur after LB formation, as pSer129 α-syn accumulation in LBs is detectable only in the late stages of DLB progression [52, 54]. Further characterization of the exosomal cargo for possible α-syn variants may further elucidate the toxicity of DLB exosomes as well as the role of pSer129 α-syn in LB formation.

Studies with synthetic α-syn proteins reported less aggregation between human α-syn and endogenous α-syn in rodent brains [33]. Although DLB exosomes contained α-syn (Figs. 3a and 5b), it was unknown at the time if the amount inside DLB exosomes would be sufficient for immunohistological detection. Aware of this caveat, we harvested the DLB and Ctl-injected brains at 4 weeks. Indeed, we detected expression of human α-syn in DLB-injected tissue with punctate colocalization with mouse α-syn (Fig. 4g, h). These data suggest the possibility of mouse and human α-syn interactions in the terminals, where α-syn typically resides in neurons [6]. Longer time points would address whether this particular expression pattern of human α-syn persists and if human α-syn is targeted by the lysosomal pathway.

Translocation of extracellular oligomeric α-syn often occurs through endocytosis [29], although it is not clear how α-syn triggers uptake. Another way exosomes could optimize α-syn internalization and therefore aggregation is by activating endocytic pathways. Indeed, sonicating exosomes disrupted α-syn internalization, suggesting that exosomes need to be intact to efficiently shuttle α-syn into the cell [11]. In addition, internalization of exosomes was reduced with the digestion of exosome surface proteins by proteases and inhibited at 4 °C [16]. This suggests that an energy dependent process such as endocytosis mediates exosome uptake. In our studies, DLB-mediated α-syn accumulation was abolished with the inhibition of endocytosis (Fig. 5). Furthermore, human α-syn highly colocalized with Rab5 in DLB exosome injected mouse brains (Fig. 4a, b). These data suggest that α-syn contained in DLB exosomes is internalized through Rab5-mediated endocytosis.

In our studies, we observed 60% DLB-derived α-syn colocalization with MAP2^+^ cells as opposed to about 2% colocalization of α-syn observed in GFAP^+^ cells (Fig. 4c-f), implying DLB exosomes express preference for neurons. Extended analysis of DLB exosome internalization in non-neuronal cells such as oligodendocyte cell lines would assess if DLB exosomes specifcially target neurons. In addition, further characterization of the subtype of the afflicted neurons would provide additional details into the pathophysiology of DLB, which may hold diagnostic relevance in discerning DLB from PD.

The article "Brain-derived exosomes from dementia with Lewy bodies propagate α-synuclein pathology" was retracted in 2026. Reasons: duplicated images; duplicated data; overlap with earlier publications; unreliable data.

## Conclusions

Exosomes are an attractive biomarker that could possibly be used to diagnose neurodegenerative diseases. Utilizing immunohistochemistry and Western blot analysis we observed that brain tissue originating from individuals diagnosed for AD or DLB (Table 1) and verified to contain α-syn, Aβ and p-Tau aggregates (Fig. 2a), produced exosomes containing elevated levels of these aggregate-prone proteins (Fig. 2a-d). In addition, our current study demonstrates that exosomes can mediate the internalization of exogenous α-syn into naïve neuronal cells through endocytosis. These data imply exosomes may play a role in α-syn pathogenesis, possibly through the seeding of toxic forms of α-syn. Possible future studies include researching how exosomes regulate α-syn transmission based on cell subtype, which could have implications in diagnosing Lewy Body disorders.

## Abbreviations

AD: Alzheimer’s Disease
APP: Amyloid precursor protein
Aβ: Amyloid-Beta
CSF: Cerebrospinal Fluid
Ctl: Control
DLB: Dementia with Lewy Bodies
DRS: Mattis Dementia Rating Scale
MAP: Microtubule Associated Protein
MCI: Mild Cognitive Impairment
MVB: Multivesicular bodies
Rab5: Ras-Related Protein 5
TEM: EM, Transmission Electron Microscopy
α-syn: α-synuclein
